The article "Sulforaphane Improves Ischemia-Induced Detrusor Overactivity by Downregulating the Enhancement of Associated Endoplasmic Reticulum Stress, Autophagy, and Apoptosis in Rat Bladder" was retracted in 2023. Reasons: duplicated images; original data or images not available; unreliable data.

# Sulforaphane Improves Ischemia-Induced Detrusor Overactivity by Downregulating the Enhancement of Associated Endoplasmic Reticulum Stress, Autophagy, and Apoptosis in Rat Bladder

**DOI:** 10.1038/srep36110

**Published:** 2016-11-08

**Authors:** Huai-Ching Tai, Shiu-Dong Chung, Chiang-Ting Chien, Hong-Jeng Yu

**Affiliations:** 1 Department of Urology, National Taiwan University Hospital and National Taiwan University College of Medicine, Taipei, Taiwan; 2 Graduate Institution of Clinical Medicine, National Taiwan University College of Medicine, Taipei, Taiwan; 3 Department of Urology, Far East Memory Hospital, New Taipei City, Taiwan; 4 Graduate Program in Biomedical Informatics, College of Informatics, Yuan-Ze University, Chung-Li, Tao-Yuan, Taiwan; 5 Department of Life Science, National Taiwan Normal University, Taipei, Taiwan

## Abstract

Atherosclerosis-associated pelvic ischemia has been reported to be a risk factor for bladder dysfunction and subsequent lower urinary tract symptoms (LUTS) in the elderly population. However, the molecular mechanisms of this association remain unclear. We hypothesized that stress-induced cellular responses might play a role in the pathogenesis of ischemia-induced bladder dysfunction. In the present study, the animal model of bladder ischemia was induced by bilateral partial arterial occlusion (BPAO) in rats. We found that BPAO significantly induced the presence of detrusor overactivity (DO) and upregulated the expression of several molecular reactions, including biomarkers in endoplasmic reticulum stress (78 kDa glucose-regulated protein, GRP78 and C/EBP-homologous protein, CHOP), autophagy (Beclin-1, p62 and LC3 II) and apoptosis (caspase 3). BPAO also disturbed the Kelch-like ECH-associated protein 1–nuclear factor erythroid-2-related factor 2 (Keap1–Nrf2) pathways. These responses might collectively alter muscarinic and purinergic signaling and contribute to the presence of DO in the ischemic bladder. Therapeutically, treatment with neither a muscarinic nor purinergic receptor antagonist restored bladder function. Interestingly, sulforaphane effectively attenuated ischemia-enhanced endoplasmic reticulum stress, autophagy and apoptosis in the bladder, subsequently ameliorated ischemia-induced bladder dysfunction and might emerge as a novel strategy to protect the bladder against ischemia-induced oxidative damage.

Several visceral organs are susceptible to ischemic injury, such as the heart, bowel, and kidneys^1^,^2^,^3^. Ischemia has also been recently postulated to be involved in the pathogenesis of non-obstructive, non-neurogenic bladder dysfunction and the subsequent development of lower urinary tract symptoms (LUTS), especially in the elderly population. A close correlation between LUTS and vascular risk factors, such as smoking and hypertension, may suggest that aging-associated pelvic atherosclerosis is a potential mechanism^4^,^5^. Similarly, our epidemiological research has also demonstrated that metabolic syndrome is a risk factor for LUTS and overactive bladder (OAB) in women with type 2 diabetes^6^. Although the underlying pathophysiology remains unclear and may be multifactorial, individuals with metabolic syndrome are likely predisposed to bladder dysfunction via atherosclerosis-induced ischemia. Furthermore, substantial evidence has been provided through the direct sonographic assessment of bladder blood flow. Compared with younger asymptomatic controls, elderly patients with LUTS apparently have lower perfusion in the bladder neck and prostate^7^. Another study showed that persistent detrusor overactivity (DO) in men after transurethral resection of the prostate is associated with an increase in the vascular resistance of bladder vessels and a subsequent reduction of perfusion and hypoxia, suggesting that chronic ischemia may also play a role in addition to bladder outlet obstruction^8^.

Although various mechanisms that involve bladder innervation, epithelium, and disproportionate increases in prostaglandin and leukotriene production have been proposed^9^,^10^,^11^,^12^, the molecular pathways that underlie ischemia-induced bladder dysfunction are still largely unknown. Excess oxidative stress secondary to ischemia/reperfusion has been reported to cause mitochondrial dysfunction and neurodegeneration, leading to bladder overactivity^13^,^14^. Another cellular organelle, the endoplasmic reticulum (ER), may also be involved in the cellular damage under conditions of oxidative stress^15^. The ER is responsible for protein synthesis and maturation and also plays a crucial role in monitoring intra- and extracellular stress. Disturbances in ER homeostasis may cause the accumulation of unfolded or misfolded proteins, resulting in ER stress^16^,^17^. ER stress has been implicated in several pathophysiological conditions^18^,^19^,^20^ and integrates multiple cellular responses, including inflammation, autophagy, and apoptosis^21^,^22^,^23^.

Nuclear factor erythroid-2-related factor 2 (Nrf2) is an inducible transcription factor that has been shown to play a critical role in cellular protection against oxidative stress. Under basal conditions, Nrf2 is bound to its cytoplasmic repressor Kelch-like ECH-associated protein 1 (Keap1), which mediates the ubiquitination of Nrf2. When there is an abundance of reactive species in the cell, the nuclear translocation of Nrf2 launches and binds to a cis-acting promoter sequence called antioxidant response element (ARE), allowing the transactivation of a group of ARE-driven detoxification and antioxidant genes. Therefore, Nrf2 activation has emerged as a promising strategy that confers resistance to various ischemic, oxidative, and inflammatory insults. The Nrf2 pathway has also been suggested to be closely associated with other stress signal cross-talk and might orchestrate the progression of some pathological conditions^14^,^24^.

We hypothesized that bladder ischemia that is induced in our experimental model might elicit oxidative stress and subsequent cellular responses, leading to bladder dysfunction. The attenuation of these stress-related alterations might alleviate damage and possibly provide insights into a novel strategy to protect against ischemia-induced bladder dysfunction.

## Methods

### Experimental Animals

Forty-eight female Wistar rats (250 g, Orient Bio, Seongnam, Korea) were housed in the Laboratory Animal Center of National Taiwan University, College of Medicine, under conditions of constant temperature and a consistent light cycle (lights on from 7:00 AM to 6:00 PM). All of the animal surgical and experimental procedures were approved by the Institutional Animal Care and Use Committee of National Taiwan University, College of Medicine and College of Public Health (approval no. 20090278), and were performed in accordance with the guidelines of the National Science Council of the Republic of China (NSC 1997). All efforts were made to minimize animal suffering and the number of animals that were used in the experiment.

### Induction of Bladder Ischemia by Bilateral Partial Arterial Occlusion (BPAO) and Drug Administration

The animal model of bladder ischemia is illustrated in Fig. 1. The rats were divided into four groups: sham control (*n* = 8), 2 weeks of ischemia (2WBI, *n* = 8), 4 weeks of ischemia (4WBI, *n* = 8), and 4WBI with treatment (*n* = 18). Under avertin anesthesia (200 mg/kg body weight, i.p.), a 12-mm incision was made on the angle of the both hind legs (inguinal area), and the femoral vessels were exposed by blunt dissection. The artery and vein were separated as one unit. A lower midline abdominal incision was then made, and the bilateral common iliac arteries bifurcating at the terminal of the abdominal aorta were exposed and carefully isolated. Polyethylene-10 (PE-10) tubing was inserted through the femoral artery into the abdominal aorta and removed freely after the common iliac artery was tied with a 3/0 silk ligature (Fig. 1B), thus enabling the artery to be partially occluded (Fig. 1C). The contralateral side was done similarly. The surgical procedure is illustrated in Fig. 1D–F. The abdominal and inguinal wounds were closed, and the rats were given ampicillin (150 mg/kg body weight, i.m.) once per week for 2 weeks. In the sham group, all of the surgical preparations and procedures were performed similarly without catheterizing the arteries.

To investigate the drugs’ effects on BPAO-induced DO, the 4WBI group was treated daily with the selective purinergic P_2_X antagonist pyridoxalphosphate-6-azophenyl-2′,4′-disulfonate (PPADS; 1 μM/kg, i.p.; Sigma, St. Louis, MO, USA; *n* = 6), muscarinic antagonist atropine (5 μM/kg, i.p.; Sigma, St. Louis, MO, USA; *n* = 6), and Nrf2 activator sulforaphane (SR; 0.7 mmoL/kg dissolved in corn oil, i.p.; LKT Laboratories, St. Paul, MN, USA; *n* = 6). The drugs were administered 1 week after the induction of bladder ischemia.

### Measurement of Bladder Microcirculation

To determine the effects of BPAO on bladder hemodynamics, a full-field laser perfusion imager (Moor FLPI, Moor Instruments, Devon, UK) was used to quantify microcirculatory blood flow intensity in the bladder in six rats. Moor FLPI allows the continuous non-contact recording of blood flow in the microvasculature in the rat bladder. This imager uses laser speckle contrast imaging, which exploits the random speckle pattern that is generated when tissue is illuminated by laser light. The random speckle pattern changes when blood cells move within the region of interest (ROI). When there is a high level of movement (fast flow), the changing pattern becomes more blurred, and the contrast in that region is reduced accordingly. Therefore, low contrast is related to high flow, and high contrast is related to low flow. The contrast image is processed to produce a 16-color-coded image that correlates with blood flow in the tissue. Blue indicates low flow, and red indicates high flow (range, 0–1000). The microcirculatory blood flow intensity in each ROI was recorded as Flux with perfusion units, which is related to the product of the average speed and concentration of moving red blood cells in the tissue sample volume. The images were recorded and analyzed in real time using Moor FLPI 3.0 software (Moor Instruments). The microcirculatory blood flow intensities were compared among the three groups at different time points.

### Evaluation of Cystometric Parameters

We utilized a transcystometric model to evaluate micturition alterations in the bladder in response to BPAO. This method has been well-established in our laboratory^25^,^26^. Briefly, the rats were anesthetized by a subcutaneous injection of urethane (1.2 g/kg body weight). After the bladder was exposed through a midline incision of the abdomen, a PE-50 catheter (bladder catheter) was inserted through the apex of the bladder dome and connected via a T-tube to a P23 ID infusion pump and pressure transducer (Gould-Statham, Quincy, MA, USA). Cystometry was performed using saline at an infusion rate of 0.04 ml/min. The intravesical pressure (IVP) was continuously recorded using an ADI system (Power-Lab/16S, ADI Instruments, Castle Hill, Australia). The following parameters of bladder responsiveness were measured: intercontraction interval (ICI; i.e., the time interval between two micturition cycles identified with active contractions [>15 mmHg]), baseline bladder pressure (BP), threshold pressure for triggering micturition (PTH), and maximal contractile amplitude (MCA).

### Measurement of Reactive Oxygen Species *In Vivo*

*In vivo* bladder reactive oxygen species (ROS) production in response to ischemia was measured directly from the bladder surface by continuous intravenous infusion of the chemiluminescence (CL) probe 2-methyl-6-(4-methoxyphenyl)-3,7-dihydroimidazo-[1,2-*a*]-pyrazin-3-one hydrochloride (MCLA; TCI-Ace, Tokyo Kasei Kogyo, Tokyo, Japan) at a dose of 4 μg/min and examined by the Chemiluminescence Analyzing System (CLA-ID3, Tohoku Electronics, Sendai, Japan)^26^. Briefly, the animals were individually housed in a dark box with a shielded plate to prevent photon emissions from other sources. The tissue window was left unshielded and positioned under a reflector that reflected the photons from the exposed tissue surface onto the detector area. The CLA-enhanced CL signal from the sample surface was continuously measured by the Chemiluminescence Analyzing System during administration. The detection of *in vivo* CL generation was performed for a total of 4 h. During the procedure, the CL measurement was stopped and resumed immediately after completing the procedure.

### Tissue Collection

After the experiments, the bladder was removed, and one part of the bladder was fixed in 4% buffered formalin for morphological staining. Part of the samples was stored at −70 °C for adenosine triphosphate (ATP) and acetylcholine (ACh) content measurement and postsynaptic receptor protein expression analysis by Western blot.

### *In Situ* Detection of Oxidative Stress, Fibrosis, Endoplasmic Reticulum Stress, Apoptosis and Autophagy

Sections (5 μm) of formalin-fixed bladders were stained with hematoxylin and eosin (H&E) for evaluation of the extent of neutrophils infiltration. We performed toluidine blue staining for specific mast cell labeling and CD68 immunostaining to evaluate monocyte/macrophage distribution in the damaged urinary bladder. In brief, tissue sections were washed with Tris-buffered saline and incubated with toluidine blue solution (Polysciences, 1 g/100 mL of 70% ethanol stock) diluted 1:10 with 1 g/mL aqueous NaCl for 2 min followed by 3 rinses with deionized water. Specific mast cell stain was demonstrated in blue color under microscopic observation. For CD68 cells (monocyte/macrophage) staining, the tissue sections were incubated overnight at 4 °C with a mouse anti-rat antibody to CD68 (F4/80, 1:200, Serotec, Sydney, Australia). Bladder sections were stained with Masson’s trichrome for evaluation of the degree of interstitial collagen deposition as described before^14^.

We also used 3-nitrotyrosine (3-NT) to evaluate the presence and distribution of oxidative stress, 78 kDa glucose-regulated protein (GRP78) and C/EBP-homologous protein (CHOP) staining to determine ER stress, Beclin-1 staining to determine autophagy, and terminal deoxynucleotidyl transferase-mediated nick-end labeling (TUNEL) to determine apoptosis in the paraffin-embedded sections of bladder tissues.

Bladder sections that were obtained from 10% formalin fixation and paraffin embedding were deparaffinized, rehydrated, and immunohistochemically stained for 3-NT by incubating them a polyclonal antibody (Alpha Diagnostic International; San Antonio, TX, USA) diluted 1:50. Brown deposits per total section area were counted by Adobe Photoshop 7.0.1 image analysis software. For GRP78, CHOP, Beclin-1 and LC3 II staining, the tissue sections were incubated overnight at 4 °C with mouse anti-rat GRP78, CHOP, Beclin-1 antibodies (BioSource International, Camarillo, CA, USA) and LC3 II antibody (Medical & Biological Laboratories, Co., Ltd., Naka-ku, Nagoya, Japan). Biotinylated secondary antibody (Dako, Botany, Australia) was then applied, followed by streptavidin conjugated to horseradish peroxidase (HRP; Dako). The chromogen was Dako Liquid diaminobenzene (DAB). The TUNEL method was performed according to a method described previously. Briefly, 5-mm thick sections of the bladder were prepared, deparaffinized, and stained by the TUNEL-ABC method.

For quantification, 10 sections from each sample were stained with specific stains. Twenty high-power (x400) fields were randomly selected for each section, and the value of neutrophils, CD68 cells, mast cells and TUNEL-apoptotic cells was counted. The percent change in 3-NT, Masson, GRP78, CHOP, Beclin-1 and LC3 II staining equals the total area of brown staining for 3-NT, Masson, GRP78, CHOP, Beclin-1 and LC3 II divided by the total area in the region of interest in the section.

### Translocation of Nuclear Nrf2

We evaluated the expression of Nrf2 and I-Nrf2 (Keap1) in the nucleus and cytosol. The isolated cortices were placed in ice-cold isolation buffer that contained 0.5 M sacarose, 10 mM Tris-HCl, 1.5 mM MgCl_2_, 10 mM KCl, 10% glycerol, 1 mM ethylenediamine tetraacetic acid (EDTA), 1 mM dithiothreitol, 2 μg/ml aprotinin, 4 μg/ml leupeptin, 2 μg/ml chymostatin, 2 μg/ml pepstatin, and 100 μg/ml 4-(2 aminoethyl)-benzenesulfonyl fluoride, pH 7.4, and homogenized using a tissue grinder^14^. The homogenate was centrifuged at 4,000 × *g* for 5 min at 4 °C to remove incompletely homogenized fragments and nuclei. The pellet was resuspended in lysis buffer and centrifuged at 12,000 × *g* for 20 min at 4 °C. The supernatant was then resuspended in isolation buffer, and the aliquots (nuclear fractions) were stored at −70 °C. We used β-actin and Lamin A/C for Western blot to normalize the cytosolic and nuclear fraction protein amounts, respectively. Hsp70 and β-actin were purchased from Sigma-Aldrich (St. Louis, MO, USA), and Nrf2, I-Nrf2, and Lamin A/C were purchased from Santa Cruz Biotechnology (Santa Cruz, CA, USA).

### Measurement of Adenosine Triphosphate and Acetylcholine Contents

The portion of the bladder above the ureteral orifices was harvested as the bladder body. Under a dissecting microscope (Olympus SZ61), the muscle layers were obtained from the bladder body wall by stripping off the urothelium and mucosa with sharp tweezers (Dumont, Switzerland). To avoid cross-contamination by these two layers, the proficiency of separation was histologically assessed as described previously^27^. We further analyzed the ATP and ACh content and postsynaptic receptor expression in the isolated smooth muscle layers. The smooth muscle layers were collected for ATP and ACh content analysis. Bladder ACh content was measured using a commercial kit (Choline/ACh Quantification Kit, K615–100, BioVision, Milpitas, CA, USA). The kit can detect 10 pmol-5 nmol of ACh. The isolated smooth muscle tissue was homogenized in Choline Assay Buffer and centrifuged at 600 × *g* for 30 min to remove debris. The supernatant was tested by mixing sufficient reagents in each well. A total of 50 μl of the reaction mixture contained 44 μl Choline Assay Buffer, 2 μl choline probe, 2 μl acetylcholinesterase, and 2 μl enzyme mixture. All of the samples were incubated at room temperature for 30 min in a dark room, and the optical density (OD) was measured at 570 nm for the colorimetric assay in a micro-plate reader (Wallac 1420 vector2, PerkinElmer, San Jose, CA, USA). We subtracted the background value (the 0 choline control) from all standard and sample readings.

Bladder ATP content was measured using a luciferin-luciferase assay kit (Roche, Penzberg, Germany) according to the manufacturer’s instructions. This method measures the ATP dependency of the light-emitting luciferase-catalyzed oxidation of luciferin. The isolated smooth muscle tissue was homogenized using liquid nitrogen and diluted in a buffer that contained 100 mM Tris and 4 mM EDTA (pH 7.75) and immediately mixed with equal amounts of luciferase reagent. The light that was emitted from the luciferase was measured using a Chemiluminescence Analyzing System (CLA-ID3, Tohoku Electronic, Sendai, Japan), and the values were calibrated against a standard ATP curve. We used an ATP Colorimetric/Fluorometric Assay Kit (catalog no. K354–100, BioVision, Milpitas, CA, USA) to further determine ATP content in the muscle layer of the urinary bladder. For the colorimetric assay, the ATP standard was prepared to obtain 0, 2, 4, 6, 8, and 10 nmol/well of ATP standard. The bladder tissue was homogenized using perchloric acid (catalog no. K808–200, BioVision, Milpitas, CA, USA) and centrifuged ice cold at 15,000 × *g* for 2 min to collect the supernatant. The supernatant was mixed with 44 μl ATP Assay Buffer, 2 μl ATP probe, 2 μl ATP converter, and 2 μl developer mix. All of the samples were incubated at room temperature for 30 min in a dark room, and the OD was measured at 570 nm for the colorimetric assay in a micro-plate reader (Wallac 1420 vector). We subtracted the background value (the 0 ATP control) from all standard and sample readings.

### Western Blot

The expression levels of the ER stress-related proteins GRP78 and CHOP, apoptosis-related protein caspase 3, autophagy-related protein Beclin-1, LC3 II and p62, muscarinic M_2_ and M_3_ receptors, and purinergic P_2_ X _1_, P_2_ X _2_, and P_2_ X _3_ receptors in bladder smooth muscle layer tissues were analyzed by Western blot as described previously^14^. The bladder smooth muscle samples were homogenized with a prechilled mortar and pestle in extraction buffer, which consisted of 10 mM Tris-HCl (pH 7.6), 140 mM NaCl, 1 mM phenylmethylsulfonyl fluoride, 1% NP-40, 0.5% deoxycholate, 2% β-mercaptoethanol, 10 mg/ml pepstatin A, and 10 mg/ml aprotinin. The mixtures were completely homogenized by vortexing and kept at 4 °C for 30 min. The homogenate was centrifuged at 12,000 × g for 12 min at 4 °C. The supernatant was collected, and the protein concentrations were determined by the BioRad Protein Assay kit (BioRad Laboratories, Hercules, CA, USA). Antibodies raised against Bax (Chemicon international Inc., Billerica, MA, USA), Bcl-2 (Transduction, Bluegrass-Lexington, KY, USA), Beclin-1 (Cell Signaling Technology, Danvers, MA, USA), LC3 II (Medical & Biological Laboratories, Co., Ltd., Naka-ku, Nagoya, Japan), p62 (Cell Signaling Technology, Danvers, MA, USA), activation fragments (32 kDa of proenzyme and 17 kDa of cleaved product) of caspase 3 (CPP32/Yama/Apopain, Upstate Biotechnology, Lake Placid, NY, USA), CHOP (L63F7, Cell Signaling Technology, Danvers, MA, USA), GRP78/Bip (Santa Cruz Biotechnology, Santa Cruz, CA, USA), M_2_ receptors (AB5166, Chemicon international Inc., Billerica, MA, USA), M_3_ receptors (Alomone Labs Ltd., Jerusalem, Israel), P_2_X_1_ receptors (Santa Cruz Biotechnology, Santa Cruz, CA, USA), P_2_X_2_ receptors (Neuromics, Northfield, MN, USA), P_2_X_3_ receptors (Santa Cruz Biotechnology, Santa Cruz, CA, USA), and β-actin (Sigma, St. Louis, MO, USA) were used. Sodium dodecyl sulfate-polyacrylamide gel electrophoresis was performed on 12.5% separation gels in the absence of urea and stained with Coomassie brilliant blue. For immunoblotting, proteins were transferred to Immobilon polyvinylidene difluoride membranes (Millipore, Billerica, MA) for 75 min at 20 V in a Miniprotean III transfer tank (Bio-Rad, Hercules, CA). Immunoreactive bands were detected by incubation with the respective antibodies described above, followed by secondary antibody-alkaline phosphatase, and finally NBT and 5-bromo-4chloro-3-indolyl phosphate, toluidine salt (Roche Diagnostic, Mannheim, Germany) stock solution for 30 min at room temperature. The density of the band with the appropriate molecular mass was semi-quantitatively determined by densitometry using an image analysis system (Alpha Innotech, San Leandro, CA, USA).

### Statistical Analysis

All data are presented as mean ± standard error of the mean (SEM). Statistically differences between data were evaluated by Student’s t-test or one-way analysis of variance (ANOVA) followed by Tukey’s post hoc test. For comparison between groups over time or other factors, a multiple-measurement ANOVA was used. A result of *P* < 0.05 was considered statistically significant. Statistical analyses were performed using SPSS 18.0 statistics software (IBM Corp., Armonk, NY).

## Results

### BPAO Induced Bladder Ischemia and Altered Cystometric Parameters

Blood pressure, bladder pressure, oxygenation, and microcirculation in response to BPAO were simultaneously measured (Fig. 2A). These statistic data showed that arterial blood pressure (Fig. 2A-1) and bladder pressure (Fig. 2A-2) remained stable before and after surgery, but bladder oxygenation (Fig. 2A-3) and blood flow (Fig. 2A-4) decreased significantly after the arteries were partially occluded.

The real-time measurements of bladder microcirculation with laser speckle contrast imaging are presented in Fig. 2B. In response to acute BPAO (Fig. 2B-b), a significant redistribution of color-coded images of ROI 2 in the bladder body (Fig. 2B-b1) associated with a decline in high-flow areas (red) and an increase in low-flow areas (blue) was observed (Fig. 2B-b3) when compared to the ROI 2 image (Fig. 2B-a1) and histogram (Fig. 2B-a3) before bladder ischemia indicating that the model of bladder ischemia was successfully induced following BPAO. Four weeks of BPAO further decreased the percentage of red-color ROI 2 image (Fig. 2B-c1) and histogram (Fig. 2B-c3). Acute BPAO and 4-week BPAO significantly decreased bladder microcirculation by the reduced perfusion units (Fig. 2B-1).

The cystometric parameters in the sham and ischemia groups are shown in Table 1. DO was characterized by a shortened ICI in the 2WBI and 4WBI groups. Additionally, the ischemic bladder was associated with a decrease in compliance, reflected by increases in BP and PTH. The MCA was also reduced in the ischemia groups.

The original cystometrograms are shown in Fig. 3. The pattern of cystometrogram in normal sham group was displayed in a slow-speed (Fig. 3A1) and fast-speed chart (Fig. 3A2). The marked phase 1 and phase 2 contractions were identified in sham group (Fig. 3A2). BPAO markedly induced DO and reduced contractile amplitude in the 2WBI (Fig. 3B1) and 4WBI groups (Fig. 3C1) in the slow-speed graphs. Furthermore, the contractile components of phase 1 and 2 in fast-speed charts changed markedly after BPAO in the 2WBI (Fig. 3B2) and 4WBI groups (Fig. 3C2).

### BPAO Increased Bladder ROS and Fibrosis

Bladder ROS levels in response to ischemia were measured by a chemiluminescent analyzer. As shown in Fig. 4A–C, ROS counts in terms of O_2_^−^, H_2_O_2_, and nitric oxide (NO) significantly increased in the 2WBI and 4WBI groups compared with the sham group. To identify the possible sources of ROS in the ischemic bladder, we evaluated neutrophils, mast cells, CD68 cells (monocyte/macrophage) infiltration, and 3-NT staining in the ischemic bladder. As shown in Fig. 5, marked increases in neutrophils (Fig. 5A–C), mast cells (Fig. 5D–F), CD68-positive cells (Fig. 5G–I), and 3-NT staining (Fig. 5J–L) were observed in the 2WBI and 4WBI groups compared with the sham group. The statistic data further showed that the level of neutrophils (Fig. 5P), mast cells (Fig. 5Q), CD68 positive cells (Fig. 5R) and 3-NT stains (Fig. 5S) was significantly higher in the 4WBI group than in the 2WBI group.

Our data also showed a significant increase in hydroxyproline content after BPAO (Fig. 4D). We evaluated the degree and distribution of bladder fibrosis by Masson’s trichrome staining. As shown in Fig. 5M–O, collagen deposition (blue staining) was markedly observed in the bladder of the 2WBI and 4WBI groups compared with the sham control bladder. The statistic data further indicated that the area of Masson stain (Fig. 5T) was significantly higher in the 4WBI group than in the 2WBI group.

### BPAO Altered Keap1-Nrf2 Signaling in the Urinary Bladder

Our data showed that under unstressed conditions, c-Nrf2 and Keap1 were maintained at low levels (Fig. 6A,B), and the modest nuclear translocation of Nrf2 (n-Nrf2; Fig. 6C) was found to maintain normal cellular homeostasis. Upon exposure to BPAO, Keap1 expression increased significantly, but n-Nrf2 levels decreased significantly, indicating that the nuclear translocation of Nrf2 was disturbed and the Keap1-Nrf2 pathway was altered by ischemic damage.

### BPAO Induced ER Stress, Autophagy, and Apoptosis in the Urinary Bladder

To investigate the role of ER stress following ischemic stress in the bladder, we examined GRP78 and CHOP expression. In the present study, substantial expression of GRP78 was observed by Western blot in the 2WBI and 4WBI groups (Fig. 6D). The expression of CHOP, a pro-apoptotic transcription factor, was significantly and time-dependently increased after BPAO (Fig. 6E), suggesting that apoptotic signals were elicited when ER function was severely impaired by ischemic insult. The appearance of GRP78- and CHOP-positive staining was observed in 2WBI (Fig. 7B,E) and 4WBI (Fig. 7C,F) bladders compared with negative staining in the sham group (Fig. 7A,D).

We also evaluated the presence of autophagy following ischemia. Western blot indicated that the expression of Beclin-1 (Fig. 6G) and LC3 II (Fig. 6I), two well-known key regulators of autophagy, was significantly enhanced and another autophagy-related protein p62 (Fig. 6H) was significantly decreased in the ischemic bladder. Together with the overexpression of GRP78, we suggest that the enhancement in Beclin-1 and LC3 II and the decrease in p62 are involved in the activation of autophagy in response to ischemia and ER stress in the bladder. Additionally, positive Beclin-1 (Fig. 7H,I,R) and LC3 II (Fig. 7K,L,S) expression was also markedly demonstrated in 2WBI and 4WBI bladder tissue compared with the respective sham group (Fig. 7G,J). The electromyography of the bladder smooth muscles from control and 4WBI showed that the existence of autophagosomes in the 4WBI bladder not in the control bladder (Fig. 8).

Caspase 3 is a crucial component of the apoptotic machinery. As shown in Fig. 6F, the expression of caspase 3 was significantly increased in the 2WBI and 4WBI groups compared with the sham group. The presence of apoptotic cells was also significantly increased in 2WBI (Fig. 7N,T) and 4WBI (Fig. 7O,T) bladders by TUNEL following ischemic damage. Together with CHOP and caspase 3 upregulation and the presence of TUNEL-positive staining in the ischemic bladder, we suggest that caspase 3-mediated apoptosis was induced if the unfolded protein response was overwhelmed by excess ER stress secondary to high loads of ischemia-related unfolded protein.

### BPAO Affected Muscarinic Cholinergic and Purinergic Signaling in the Urinary Bladder

As shown in Fig. 9A,B, BPAO significantly depressed the levels of ACh and ATP in bladder smooth muscle in the 2WBI and 4WBI groups. These alterations were both time-dependent. To further understand the effects of BPAO on bladder neurotransmission, we evaluated the expression of muscarinic cholinergic and purinergic receptor proteins in bladder smooth muscle layers by Western blot. Compared with the sham group, the expression of muscarinic M_2_ and M_3_ receptors was significantly increased in 2WBI and 4WBI bladders (Fig. 6J,K). Similarly, significant upregulation of purinergic P_2_X_1_, P_2_X_2_, and P_2_X_3_ receptors was found in the 2WBI and 4WBI groups compared with the sham group (Fig. 6L–N).

### Administration of Nrf2 Activator Attenuated BPAO-Induced ER Stress, Autophagy and Apoptosis in the Urinary Bladder

We examined the effects of potential therapeutic agents for OAB, including the muscarinic antagonist atropine, selective purinergic P_2_X antagonist PPADS, and Nrf2 activator SR, on BPAO-induced cellular responses. As shown in Fig. 6, muscarinic and purinergic receptor antagonists did not have any beneficial effects on BPAO-induced Keap1-Nrf2 signaling alterations or the expression of GRP78, CHOP, Beclin-1, p62, LC3 II or caspase 3 in the ischemic bladders. However, SR administration significantly increased the nuclear accumulation of Nrf2 (Fig. 6C) and decreased Keap1 protein expression. Interestingly, SR also significantly reduced BPAO-induced GRP78, CHOP, Beclin-1, LC3 II and caspase 3 expression and recovered p62 expression in the bladder (Fig. 6D–I).

### Administration of Muscarinic Antagonist, Purinergic Antagonist, and Nrf2 Activator Attenuated BPAO-Induced Upregulation of Muscarinic and Purinergic Receptors in the Urinary Bladder

We also evaluated the effects of the aforementioned agents on the BPAO-induced upregulation of muscarinic receptors and purinergic receptors. As shown in Fig. 6J,M, administration of the muscarinic antagonist, the purinergic antagonist, and SR attenuated the upregulation of M_2_ and M_3_ receptors following bladder ischemia. Similar effects were observed for purinergic signaling, in which treatment with these agents effectively restored the BPAO-induced expression of P_2_X_1_, P_2_X_2_, and P_2_X_3_ receptors (Fig. 6L–N).

### Administration of Nrf2 Activator but not Muscarinic/Purinergic Antagonists Ameliorated BPAO-Induced DO in the Urinary Bladder

The effects of therapeutic agents on ischemia-induced bladder dysfunction are shown in Table 1 and Fig. 3D–F. Neither muscarinic antagonist atropine (Fig. 3D1) nor purinergic antagonist PPADS (Fig. 3E1) ameliorated BPAO-induced DO. In addition, in the fast-speed charts, the dysregulated phase 1 and 2 contractions in 4WBI rats were not effectively rescued by atropine (Fig. 3D2) or PPADS (Fig. 3E2). Moreover, these two antagonists appeared to exacerbate bladder dysfunction after 4WBI injury. The use of Nrf2 activator SR effectively ameliorated BPAO-induced DO (Fig. 3F1) and partly recovered phase 1 and 2 contractile elements in 4WBI rats (Fig. 3F2), indicating that SR was able to protect the urinary bladder against ischemic injury.

## Discussion

The present study provided evidence of the involvement of ER stress, autophagy, and apoptosis in the bladder upon BPAO injury. We found that these adaptive cellular responses were activated under conditions of ischemic stress, indicating that the bladder underwent a dynamic process that involved cytoprotective autophagy and cytodestructive apoptosis, possibly depending on the severity of ischemia in different affected areas. The induction of autophagy is crucial for the intracellular generation of amino acids, ATP, and other nutrient molecules that support cellular survival in the ischemic bladder. However, if ischemia produces excessive and prolonged ER stress and cannot be alleviated by the unfolded protein response, then pro-apoptotic signaling is triggered to cause cell suicide. Increases in ER stress, autophagy and apoptosis that are associated with the increase in oxidative stress have also been reported in other types of ischemia/reperfusion tissues^14^,^28^.

We also examined the expression of Keap1-Nrf2 signaling in the ischemic bladder, which is the major regulator of cytoprotective responses against oxidative stress. In the present study, we observed a significant decrease in the nuclear accumulation of Nrf2 in the rat bladder upon 2- and 4-week BPAO, suggesting that the subsequent Nrf2-mediated cytoprotective response might also be downregulated. This finding can be explained by the involvement of p62 protein (also known as sequestosome 1 [SQSTM1]) in the cross-talk between the Nrf2-Keap1 pathway, autophagy, and apoptosis. p62 is a multifunctional scaffold protein that acts as an adaptor for ubiquitinated proteins in selective autophagy and also becomes the substrate for degradation. Two mechanisms of Nrf2 regulation have been indicated as following. Under normal conditions, Nrf2 protein is maintained at a low level through Cul3-Keap1 targeted ubiquitination followed by proteasomal degradation. In BPAO conditions that bring about oxidative stress, p62 binds damaged cellular components, including ubiquitinated proteins, and is subsequently phosphorylated on S349. This phosphorylation enables p62 to bind with high affinity to the Keap1-Nrf2 complex and this inhibits the ability of Keap1 to ubiquitinate Nrf2. p62-Keap1-ubiquitnated protein complexes are degraded by selective autophagy and this allows Nrf2 to accumulate and translocate to the nucleus. On the other hand, Keap1-Nrf2 complexes can also be disrupted by oxidative modification of cysteine residues in Keap1 causing release of Nrf2. We suggest that a combination of these two mechanisms could happen in our experimental data. In support of the former mechanism, a reduction in p62 levels by BPAO is consistent with p62 degradation by selective autophagy following oxidative stress (Fig. 6H). It could then be postulated that a reduction in p62 levels does not result in reduced Keap1 levels here because binding and degradation might be dependent on Keap1 being in complex with Nrf2. In support of a role for the latter mechanism - the high overall Keap1 levels by BPAO seen in Fig. 6B might not necessarily lead to a decrease in overall levels of Nrf2 (Fig. 6A) because cysteines in the Keap1 binding domain could be modified by oxidation. It is suggested that further experimentation would be needed to investigate this possibility. One reason that could be proposed for this combinatorial effect is the extended duration of the experiment, and indeed the clinical situation compared to many previous studies. On the other hand, the Nrf2 response may also be counteracted by the p53-dependent apoptotic pathway if the scavenging machinery is overwhelmed by oxidative stress at a critical threshold^29^.

Another interesting finding in the present study was the alterations in muscarinic and purinergic receptor neurotransmission in the ischemic bladder. The level of ACh, the most important neurotransmitter that mediates bladder contractions, significantly decreased after the induction of ischemia in the bladder. This change was likely secondary to impaired ACh synthesis by the depression of choline acetyltransferase activity after ischemia^30^ or impaired release because of local hypoxia, leading to the compensatory upregulation of both M_2_ and M_3_ receptor expression to maintain normal bladder contractility. The overexpression of muscarinic receptors was suggested to cause DO and might be one of the potential etiologies of ischemia-induced bladder dysfunction. Moreover, we also evaluated purinergic signaling pathways, including neurotransmitter levels and receptor expression, in the bladder under ischemic pathophysiological conditions. Nutrient deprivation and mitochondrial dysfunction following ischemia and oxidative stress appeared to disrupt ATP generation, to decrease ATP levels and possibly to upregulate the purinergic receptors expression in the bladder smooth muscles. We speculate that the depletion of ATP may affect the efferent control of detrusor muscle excitability through P_2_X_1_ receptor upregulation and may alter bladder sensation via the activation of P_2_X_2_ and P_2_X_3_ receptors on sensory afferent neurons. According to our present data, these events could be co-incident but not co-dependent in the BPAO bladders.

Based on the aforementioned evidence, we found that ischemia-induced bladder dysfunction was associated with the presence of ER stress, autophagy, apoptosis, Nrf2-Keap1 signaling alterations, muscarinic receptor and purinergic receptor overexpression. However, it is unclear whether an interplay exists between these adaptive cellular responses and the regulation of bladder neurotransmission. A recent study reported that the activation of muscarinic signaling may mediate the regulation of autophagy and play a role in cardioprotection during ischemic heart disease^31^. The stimulation of muscarinic receptors has also been shown to mediate the anti-apoptotic pathway, providing substantial protection from DNA damage, oxidative stress, and impaired mitochondrial function that may be encountered in several diseases^32^,^33^,^34^. Therefore, the activation of muscarinic signaling in the bladder under conditions of ischemic stress might be a double-edged sword that triggers both pro-survival autophagy and anti-apoptotic axes to provide protective tolerance against ischemia-related damage. We suggest that the overexpression of muscarinic receptors may be co-incident with BPAO induced bladder dysfunction.

Currently, the mainstay for the pharmacological treatment of DO is muscarinic antagonists because bladder innervation is predominantly cholinergic^35^,^36^. Under some pathophysiological conditions, purinergic nerve-mediated contractions of the bladder increase by 40%, indicating that purinergic signaling may also be a novel therapeutic target for DO^37^,^38^. Interestingly, we found that chronic administration of the muscarinic antagonist significantly downregulated the expression of both muscarinic and purinergic receptors in the ischemic bladder, suggesting cross-talk between muscarinic and purinergic signaling. Similar effects were also observed with purinergic antagonist treatment. However, despite effectively restoring bladder neurotransmission following ischemic injury, neither agent ameliorated ischemia-induced bladder dysfunction. Treatment with SR, a naturally occurring isothiocyanate that is obtained from cruciferous vegetables, significantly increased the nuclear translocation of Nrf2 in the ischemic bladder and might contribute to the induction of antioxidant phase II enzymes, such as thioredoxin reductase-1, glutathione reductase, and NAD(P)H:quinone oxidoreductase^39^,^40^. The mechanism of Nrf2 activation by SR involves direct and specific Keap1 modification in the Kelch domain, leading to the dissociation of Nrf2 from Keap1^28^. Indirectly, SR also negatively regulates p38 MAP kinase, which suppresses Nrf2 activation by promoting Nrf2 phosphorylation and its interaction with Keap1^41^. Through Nrf2 activation, SR protected the bladder against ischemia-induced oxidative damage by attenuating the presence of associated ER stress, autophagy, and apoptosis. Moreover, SR downregulated the expression of muscarinic and purinergic signaling in the ischemic bladder. However, in contrast to the muscarinic and purinergic antagonists, which failed to ameliorate ischemia-induced DO, SR effectively modified bladder function following BPAO by restoring bladder compliance and contractility. The reason for this difference is not yet clear, but we purpose that alterations in bladder neurotransmission alone are unable to explain the full spectrum of ischemia-induced DO. Other molecular mechanisms that result from BPAO injury might also contribute to the development of ischemia-induced DO, suggesting that the blockade or downregulation of bladder signaling pathways was not sufficiently effective to reduce the extent of ischemia-induced DO because neither treatment protected the bladder from persistent and cumulative oxidative stress secondary to BPAO, as shown in the present study. Therefore, the upstream attenuation of cellular responses through Nrf2 activation might emerge as a therapeutic strategy to treat ischemia-induced bladder dysfunction. The hypothetical mechanism of ischemia-induced DO is illustrated in Fig. 10.

On the other hand, many diseases involve combinations of oxidative stress (Nrf2 activation), low oxygen tension (hypoxia-induced factor-1α, HIF-1α activation), and inflammatory responses (NF-κB activation). HIF-1α expression is not only associated with tumorigenesis and angiogenesis, but is also found in mammalian cells growing at low oxygen concentrations and as a consequence of ischemia/reperfusion injury^42^. Ischemia/reperfusion enhanced HIF-1α, inducible nitric oxide synthase (iNOS) and caspase 3 expression^43^. SR is an effective chemopreventive compound for Nrf2 activation against ischemia/reperfusion induced cardiomyocytes injury through the increase of survival rate and the decrease of iNOS, HIF-1α and caspase 3 expression^43^. SR also confers anticarcinogenic, antiproliferative and antioxidant activities to induce deleterious changes in cancer cell mitochondria that eventually would carry the cell to death via apoptosis and to protect noncancer cell mitochondria against oxidative challenge, which prevented cell death^44^. The use of a novel strategy to study simultaneous activation of Nrf2, HIF-1α, and NF-κB in single cells found that upon challenges of cells with several redox-perturbing conditions, Nrf2, HIF-1α, and NF-κB are uniquely responsive to separate stimuli, but can also display marked cross talk to each other within single cells^45^. Cumulated evidence indicated that in addition to Nrf2 activation, SR can be a histone deacetylase inhibitor, aryl hydrocarbon receptor nuclear translocator inhibitor/repressor, HIF-1α repressor and HSF1 activator^46^,^47^,^48^. It is still uncertain how SR changes the response in Nrf2 regulation system. A possible mechanism put forward by Keum^49^ is that a number of putative kinases are reported to directly phosphorylate the Nrf2 protein and affect its cellular location or stability. Although it is still uncertain whether ERK and JNK can directly phosphorylate the Nrf2 protein, there are a significant number of papers showing that SR is a strong inducer of ERK and JNK phosphorylation and that these two signaling kinases are critically involved in the activation of ARE-dependent gene expression. All the above messages suggest that in addition to Nrf2 activation, SR may also provide alternate mechanisms to protect against ischemic/hypoxic injury.

In conclusion, the present study found that BPAO significantly induced the DO associated with the presence of GRP78/CHOP-mediated ER stress, Beclin-1/p62/LC3 II-related autophagy, caspase 3-mediated apoptosis, and Keap1-Nrf2 signaling disturbances in the bladder. BPAO also led to alterations in bladder neurotransmission and possibly contributed to the development of ischemia-induced DO. Treatment with the SR but not a muscarinic or purinergic antagonist effectively improved ischemia-induced bladder dysfunction.

## Additional Information

**How to cite this article**: Tai, H.-C. *et al*. Sulforaphane Improves Ischemia-Induced Detrusor Overactivity by Downregulating the Enhancement of Associated Endoplasmic Reticulum Stress, Autophagy, and Apoptosis in Rat Bladder. *Sci. Rep.* **6**, 36110; doi: 10.1038/srep36110 (2016).

**Publisher’s note:** Springer Nature remains neutral with regard to jurisdictional claims in published maps and institutional affiliations.

## Figures and Tables

**Figure 1:** Illustration of animal model of bladder ischemia. (**A**) Arterial supply of the bladder in rats. (**B**) The CIA was tied with a 3/0 silk ligature after PE-10 tubing was inserted through the FA. (**C**) Bladder blood flow decreased after partial occlusion by tubal ligation. (**D**–**F**) Experimental photos of the animal model before (**D**), during (**E**), and after (**F**) surgery. Yellow arrows indicate the partial arterial constriction. CIA, common iliac artery; IIA, internal iliac artery; FA, femoral artery.

**Figure 2:** (**A**) Representative recordings of changes in arterial blood pressure, bladder pressure, oxygenation, and blood flow in response to bladder ischemia. (**A-1**) Statistic data of the arterial blood pressure (ABP), bladder pressure (BP), bladder oxygenation (BO) and bladder blood flow (BBF) before and after bladder ischemia by partially common iliac artery ligation (BPAO). (**B**) Laser speckle contrast analysis of relative bladder microcirculation in response to bladder ischemia. Normal bladder blood flow is shown in flux image (left), photo image (middle), and perfusion histogram of ROI 2 (right). The distribution of bladder blood flow was significantly altered after the induction of ischemia, with a decrease in the high-flow area (red) accompanied by an increase in the low-flow area (blue). Three ROIs were established: ROI 1 (right femoral artery), ROI 2 (bladder body), and ROI 3 (left femoral artery). (**B-1**) Statistic data of the ROI 2 value displayed with blood perfusion unit in red color in the three groups of rats; before BPAO, acute BPAO and 4 weeks of BPAO. *p < 0.05, compared with sham treatment (before BPAO); ^#^*p* < 0.05, compared with acute BPAO.

**Figure 3:** Representative recordings of changes in cystometrograms in the sham, 2WBI, and 4WBI groups. (**A**) Sham. (**B**) 2WBI. (**C**) 4WBI. (**D**) 4WBI plus muscarinic antagonist (MA, atropine) treatment. (**E**) 4WBI plus purinergic antagonist (PA, PPADS) treatment. (**F**) 4WBI plus Nrf2 activator (SR) treatment. 1, type 1 contraction; 2, type 2 contraction. The left panel shows slow-speed charts. The right panel shows fast-speed charts that are indicated by asterisks (*) in the slow-speed charts.

**Figure 4:** Bladder ROS and hydroxyproline content in response to chronic partial bladder ischemia. Changes in bladder (**A**) O_2_^−^, (**B**) H_2_O_2_, (**C**) NO, and (**D**) hydroxyproline content in response to 2WBI, 4WBI and treatments are shown. *p < 0.05, compared with sham group; ^#^*p* < 0.05, compared with 2WBI group; ^a^*p* < 0.05, compared with 4WBI + MA group; ^b^*p* < 0.05, compared with 4WBI + PA group.

**Figure 5:** Changes in oxidative stress markers and fibrosis in response to chronic partial bladder ischemia. (**A**–**C**) Neutrophils infiltration by H&E stain. (**D**–**F**) Mast cells by toluidine blue stain. (**G**–**I**) CD68 positive stains. (**J**–**L**) 3-NT staining (arrows indicate strong staining for 3-NT in the ischemic bladder). (**M**–**O**) Masson staining (arrows indicate fibrosis with blue staining). All images are magnified with x400. The scale bar is 50 μm. Respective statistic data are shown in (**P**) number of neutrophils, (**Q**) number of mast cells, (**R**) number of CD68 positive cells, (**S**) percentage of 3-NT and (**T**) percentage of Masson stain (n = 8 in each test) in each group. *p < 0.05, compared with sham group; ^#^*p* < 0.05, compared with 2WBI group.

**Figure 6:** Changes in bladder expression of (**A**) c-Nrf2, (**B**) Keap1, (**C**) n-Nrf2, (**D**) GRP78 (ER stress), (**E**) CHOP (ER stress), (**F**) caspase 3, (**G**) Beclin-1, (**H**) p62, (**I**) LC3 II, (**J**) muscarinic M_2_ receptor, (**K**) muscarinic M_3_ receptor, (**L**) purinergic P_2_X_1_ receptor, (**M**) purinergic P_2_X_2_ receptor, and (**N**) purinergic P_2_X_3_ receptor in response to 2WBI, 4WBI, and treatments. All of the experiments were performed in three rats of each group. *p < 0.05, compared with sham group; ^#^*p* < 0.05, compared with 4WBI group; ^a^*p* < 0.05, compared with 4WBI + MA group; ^b^*p* < 0.05, compared with 4WBI + PA group.

**Figure 7:** Representative histological findings in response to bladder ischemia. The figure shows (**A**–**C**) GRP78 staining, (**D**–**F**) CHOP staining, (**G**–**I**) Beclin-1 staining, (**J**–**L**) LC3 II, and (**M**–**O**) TUNEL staining in the sham, 2WBI, and 4WBI groups. All images are magnified with x400. The scale bar is 50 μm. Respective statistic data are shown in (**P**) GRP78, (**Q**) CHOP, (**R**) Beclin-1, (**S**) LC3 II and (**T**) TUNEL stain (n = 6 in each test) in each group. *p < 0.05, compared with sham group; ^#^*p* < 0.05, compared with 2WBI group.

**Figure 8:** Electron micrography reveals bladder smooth muscle in the control (Con) animals and four weeks of BPAO animals (4WBI). (**A**) no autophagosomes were noted in bladder smooth muscle cell in Con group. (**B**) Autophagosomes (arrows) were observed in bladder smooth muscle cell in 4WBI rats with DO.

**Figure 9:** Responses of micturition-related neurotransmitter levels in the sham, 2WBI, and 4WBI groups. (**A**) Acetylcholine (ACh). (**B**) Adenosine triphosphate (ATP). *p < 0.05, compared with sham group.

**Figure 10:** Schematic illustration of the hypothetical mechanism of ischemia-induced detrusor overactivity.

**Table 1:** Baseline and experimental cystometric parameters of ICI, PTH, BP and MCA in the sham, 2WBI and 4WBI groups.

Grouping	ICI (sec)	PTH (mmHg)	BP (mmHg)	MCA (mmHg)
Sham (n = 8)	152 ± 21	9.4 ± 0.8	8.8 ± 1.1	22 ± 3.0
2WBI (n = 8)	79 ± 10*	12.8 ± 1.1*	14.2 ± 1.2*	15 ± 2.9*
4WBI (n = 8)	65 ± 7.3*	14.7 ± 1.3*	15.1 ± 1.4*	12 ± 2.4*
4WBI + MA (n = 6)	55 ± 6.2*	15.6 ± 1.4*	15.9 ± 1.3*	7.4 ± 1.7*
4WBI + PA (n = 6)	58 ± 5.5*	14.5 ± 1.6*	14.8 ± 1.2*	8.8 ± 1.9*
4WBI + SR (n = 6)	105 ± 15*,#,a,b	12.1 ± 1.0*	12.3 ± 1.0*,#,a	17.4 ± 2.4*,#,a,b

^*^p < 0.05, compared with sham group; ^#^*p* < 0.05, compared with 4WBI group; ^a^*p* < 0.05, compared with 4WBI + MA group; ^b^*p* < 0.05, compared with 4WBI + PA group.
